# Effects of Exosomal microRNAs on Oral Mucosal Epithelial Cells Cocultured with Limbal Niche Cells

**DOI:** 10.1155/2022/9794950

**Published:** 2022-08-16

**Authors:** Xiaoyu Guo, Yuting Xiao, Amin Xu, Chaoye Duan

**Affiliations:** ^1^Eye Center, Renmin Hospital of Wuhan University, Wuhan 430000, China; ^2^Department of Ophthalmology, Union Hospital, Tongji Medical College, Huazhong University of Science and Technology, Wuhan 430000, China

## Abstract

Autologous cultivated oral mucosal epithelial transplantation (COMET) is an important method for the treatment of limbal stem cell deficiency (LSCD), but the appearance of peripheral corneal neovascularization after COMET has prevented its widespread use in clinical practice. Using limbal niche cells (LNCs) as feeders in the process of coculturing could inhibit the postoperative corneal neovascularization. However, the specific mechanism is still unclear. In this study, LNCs were used as feeder cells to alter the phenotype of cultured oral mucosal epithelial cells (COMECs) by mimicking the primitive limbal microenvironment. The high-throughput sequencing of COMECs cocultured with LNCs or 3T3 cells (named LNCs group and 3T3 groups) was performed, and differential miRNA expression was analyzed. A total of 99 known and 1 newly predicted miRNAs were significantly upregulated in the LNCs group, while 101 known and 8 newly predicted miRNAs were significantly downregulated. A total of 3000 target genes with the 60 most significantly differentially expressed miRNAs were predicted, and 7 upregulated and 7 downregulated miRNAs were ultimately screened. The supernatants obtained from both cocultures were found to be rich in exosomes, indicating that the intercellular communication between COMECs and LNCs or 3T3 cells was highly active. Furthermore, the expression levels of rno-miR-200-5p, rno-miR-204-5p, rno-miR-126a-3p, rno-miR-192-5p, rno-miR-211-5p, rno-miR-143-3p, and rno-miR-184 were significantly higher in the LNCs group compared to the 3T3 group, and the expression levels had a similar trend in exosomes. Meanwhile, sequencing of the cell lines revealed 7 miRNAs that were significantly downregulated in the LNCs group. Interestingly, in that case, rno-miR-23a-3p, rno-miR-379-5p, and rno-miR-127-5p were also significantly downregulated in the exosomes. In summary, this study suggested that signal transduction between cells mediated by exosomal miRNAs may be an important factor for the inhibition of angiogenesis by LNCs nourished COMECs.

## 1. Introduction

Autologous cultivated oral mucosal epithelial transplantation (COMET) is an important way for the treatment of limbal stem cell deficiency (LSCD), but the appearance of peripheral corneal neovascularization after COMET hinders its wider application in clinical practice. Several studies have demonstrated that a disruption in the balance between ocular surface proangiogenic and antiangiogenic factors mediate the neovascularization of the corneal periphery after COMET. However, the exact mechanism remains unclear. [1–3]. A previous in vitro study reported that the rate of clone formation was higher in corneal limbal epithelial cells cocultured with trophoblast cells than in those without trophoblast cells [4]. Therefore, the use of trophoblast cells may be crucial for culturing epithelial cell sheets. When cocultured with 3T3 cells, cultured oral mucosal epithelial cells (COMECs) expressed fewer antiangiogenic factors but more proangiogenic factors than that of cultured corneal epithelial cells, and this may play a crucial role in corneal neovascularization after COMET surgery [1, 5, 6]. Cells with mesenchymal stem cell phenotype in the limbus, namely, limbal niche cells (LNCs), have been successfully isolated and cultured [7]. LNCs support the proliferation and differentiation of corneal epithelial stem cells in vitro [8]. In addition, a coculture system of LNCs and oral mucosal epithelial cells (OMECs) in the early stage has been successfully established, and it has been found that LNCs could inhibit the ability of COMECs to induce angiogenesis [9]. Furthermore, in vivo studies with animal models confirmed that COMECs nourished by LNCs could inhibit peripheral corneal neovascularization and maintain normal corneal phenotype after transplantation [10, 11].

Recent studies suggest that the stability of cell phenotypes is closely related to the regulation of noncoding RNA in cocultured cells [12]. MicroRNAs (miRNAs) are noncoding single-stranded RNAs approximately 22 nucleotides long that function as important genetic regulatory elements. miRNAs regulate the speed of messenger RNA (mRNA) translation by binding to the untranslated region of the target mRNA. In addition, miRNAs regulate the expression level after gene transcription by rapidly degrading or blocking the target mRNA [13, 14]. Over the past decade, miRNAs have emerged as important regulatory molecules of gene expression in humans and other organisms, expanding the strategies available for the diagnosis and management of various diseases. Under physiological conditions, miRNAs play key roles in controlling tissue homeostasis and cell signaling and function as posttranscriptional regulators of gene expression. The coordinated functions of these molecules are associated with other mechanisms that prevent abnormal cell proliferation, regulate cell differentiation, and respond to detected endocrine hormones and other stimuli, such as cytokines, chemokines, and infectious or stressful conditions; miRNAs are finely regulated and control the expression and function of more than 60% of the proteins in humans [15]. Several studies have reported that miRNAs, such as miR-92a, modulate neovascularization by inhibiting the expression of the integrin-*α*5 pathway, thereby inhibiting new blood vessel formation [16]. Similarly, miR-93 prevents angiogenesis by inhibiting multiple genes and signaling pathways, such as P21, E2F1, integrin-*β*8, and LATS2 [17].

In this study, high-throughput sequencing of the COMECs coculture with 3T3 cells (named 3T3 group) and LNCs (named LNCs group) was performed, and the differences between the two were analyzed using bioinformatics. Through target gene prediction and metabolic pathway analysis, the miRNA-mRNA network regulatory pathways related to angiogenesis were mined, and the mechanism by which coculture of LNCs and COMECs inhibits neovascularization was identified. In addition, the exosomal miRNAs in the cocultured cell supernatants were verified by quantitative reverse transcription polymerase chain reaction (RT-qPCR), indicating that in the coculture system, these miRNAs perform important intercellular regulatory functions and inhibit angiogenesis via exosomes.

## 2. Materials and Methods

### 2.1. Animal Materials

Healthy Sprague-Dawley (SD) rats (random sex, body weight, 200 g) were purchased from the Laboratory Animal Center of Wuhan University. The feeding and experimental operation of animals in this study were strictly in accordance with the ARVO statement and approved by the Institutional Animal Care and Use Committee at Tongji Medical College, Huazhong University of Science and Technology (IACUC number: S641). The rats were euthanized by excessive anesthesia with sodium pentobarbital, and sterile saline was injected beneath the oral mucosa. The mucosa and underlying fascia were separated, and the buccal mucosa was cut with scissors. The lateral eyeball was completely removed for subsequent cell extractions.

### 2.2. Cell Isolation and Culture

The eyeball was dissected, and the sclera and posterior segment tissue beyond 1 mm behind the limbus were removed. Limbal tissue pieces were digested with 1 mg/mL collagenase A (Roche, Indianapolis, IN, USA) for 18 h at 37°C followed by 0.25% trypsin-ethylenediaminetetraacetic acid solution (Gibco, Grand Island, NY, USA) for 20 min at 37°C to cell suspension. The cell suspension was then centrifuged with 500 g/min for 10 minutes at room temperature and the pellet was resuspended in modified embryonic stem cell medium. The cells were passaged upon reaching more than 80% confluency. When the sequential culture reached the third passage, the cells were purified, and the limbal stromal microenvironment cells (LNCs) were obtained.

Oral mucosal tissue was dispersed in 10 mg/mL Dispase II (Roche, Indianapolis, IN, USA) and digested at 37°C for 30 min. Subsequently, the epithelial cell layer was carefully torn-off with tweezers, cut into small pieces, and digested with 0.25% trypsin-EDTA solution at 37°C for 20 min to obtain a single OMEC suspension. The OMEC cell suspension was inoculated into a polyester (PET) membrane cell culture chamber (Corning, MA, USA) and cocultured with inactivated LNCs or 3T3 cells (American type culture collection). Both culture systems were cultured in keratinocyte growth medium 2 (PromoCell, Heidelberg, Germany). When the epithelial cells were substantially confluent, the volume of the medium was reduced to allow the air-lifting culture to form a stratified structure.

### 2.3. Small RNA Library Construction and Sequencing

According to the manufacturer's instructions, the total RNA of COMECs cocultured with LNCs or 3T3 cells was extracted with the QIAamp Viral RNA Mini Kit (Qiagen, Duesseldorf, Germany). Small RNA libraries were generated using the NEBNext® Multiplex Small RNA Library Prep Set (NEB, USA) following the manufacturer's recommendations. In brief, libraries were prepared by ligating different adaptors, followed by reverse transcription, PCR amplification, and size selection using 6% polyacrylamide gels. Library quality was assessed using the Agilent Bioanalyzer 2100 system, and the range of insert size was between 200 and 300 bp (Agilent, Santa Clara, CA, USA). Sequencing was performed by Bioacme Biotechnology Co., Ltd. (Wuhan, China) using Illumina Nova6000 with SE50 (Illumina, San Jose, CA, USA).

### 2.4. miRNA Analysis

Using the data quality control software Fastp V0.20, the sequencing data were filtered to filter out adapter sequences, low-quality reads (more than 40% of the reads with a base quality value below 15), and short reads (reads with a length of less than 18 nt) contaminating sequences (“N” number of reads greater than 5), clean reads were obtained, and finally 9.7–18.2 million clean reads were obtained. The clean reads were de-redundant using miRDeep2 (https://www.osc.edu/book/export/html/4389), and then, BowTie was used to map small RNA reads to the reference genome. The mapped reads were aligned with rat miRNA sequences in the miRBase database (V22) [18]. Then, the miRNA expression was counted by miRDeep2, and RPM (reads per million mapped reads) was used to normalize the miRNA expression. The differential expression analysis of miRNA was performed using DESeq2 [19]. The screening criteria for significantly different genes were corrected, *P* values of <0.05 and log2 (fold change) ≥ 1. miRNA target prediction was performed using TargetScan, PicTar, microT, miRmap, RNA22, PITA, and miRanda. The target genes were functionally annotated and enriched according to the predicted results by clusterProfiler package [20].

### 2.5. miRNA-mRNA Regulatory Network Construction

The target gene prediction of differentially expressed miRNAs was performed using miRanda software and the starBase database (V2.0) (starbase.sysu.edu.cn/index.php), which provides the prediction results of 7 miRNA databases. The target gene was predicted based on the complementarity and thermal stability of the miRNA sequence and the mRNA 3′-UTR sequence. The screening conditions were as follows: predicted score greater than 140, binding free energy less than −20 kcal/mol, and prediction by more than 1 database. The characterization of the exosomes was obtained using a similar method as previously reported [21].

### 2.6. Kyoto Encyclopedia of Genes and Genomes (KEGG) and Gene Ontology (GO) Pathway Enrichment Analyses

The biological pathway enrichment analysis based on the Kyoto Encyclopedia of Genes and Genomes (KEGG) database was performed on the differentially expressed gene set, and the significantly enriched pathways of the differentially expressed genes were extracted. The differentially expressed genes were aligned with the protein sequences in the UniProt database, and then, the alignment results were annotated by GO function according to the GO annotations in the UniProt database. We adopted the clusterProfiler package of *R* for the KEGG and GO enrichment analyses. The pathways significance was tested using hypergeometric distribution, and a *P* value of <0.05 was regarded as to be statistically significant.

### 2.7. Characterization of the Exosomes Using Electron Microscopy, Nanoparticle Analysis, and Western Blotting

The supernatants of LNCs and 3T3 groups were transferred to a clean 1.5 mL tube separately and centrifuged at 300 × *g* for 10 min and 2000 × *g* at 4°C for 20 min to remove cells and debris. Then, the exosomes were separated using the exoEasy Kit (Qiagen, Duesseldorf, Germany) and resuspended in 1 mL of PBS. The method used for the isolation of exosomes is PEG precipitation. Although there are impurities, most of the impurities are proteins, which will not affect the subsequent extraction of exosome RNA. In addition, the isolation of exosomes by ultracentrifugation requires more cell supernatant, and the cell supernatant in this study was isolated in a coculture system, which cannot meet the requirements of ultracentrifugation. According to the manufacturer's instructions, their morphological features were observed using a transmission electron microscope (H-7650; Hitachi, Japan). In addition, high-sensitivity flow cytometry for nanoparticle analysis was performed according to the manufacturer's instructions. The supernatant was collected, and the total protein concentration was determined using a bicinchoninic acid (BCA) protein assay kit (GLPBIO, Shanghai, China). Samples containing equal amounts of protein (50 *μ*g) were separated by sodium dodecyl sulphate-polyacrylamide gel electrophoresis (SDS-PAGE) and transferred onto polyvinylidene fluoride (PVDF) membranes (Millipore, Billerica, MA, USA). Protein bands were visualized with Pierce ECL Western Blotting Substrate (Thermo Fisher Scientific, Waltham, MA, USA) and exposed to an *X*-ray film.

### 2.8. RT-qPCR of Exosome miRNAs

Total RNA isolated and purified from the cell culture-exosome samples was reverse transcribed to cDNA using the miRNA RT-qPCR TB Green® Kit (TaKaRa, Dalian, China). Primer 5 was used for primer design, and all primer sequences are given in Table 1. The designed primers were synthesized by Ribobio Co., Ltd. (Guangzhou, China). The qPCR conditions were the following: 95°C for 30 s, 40 cycles at 95°C for 30 s and 60°C for 30 s; and 45 cycles at 95°C for 5 s and 60°C for 5 s. Gene expression levels were calculated by the ΔΔCt method using U6 expression as the internal control for miRNA.

### 2.9. Statistical Analysis

Statistical Product and Service Solutions (SPSS) software (version 22.0; SPSS, Chicago, IL, USA) and GraphPad Prism 8.0 (GraphPad software, San Diego, CA, USA) were used for data analysis. The data were obtained after triplicated experiments and expressed as mean ± standard deviation. The *t*-test was used to evaluate differences between groups, and a *P* value of <0.05 was regarded as to be statistically significant.

## 3. Results

### 3.1. Isolation of OMECs and Coculture with Feeder Cells

Single-cell suspensions of OMECs were cocultured in in vitro. As nonadherent cells were aspirated during medium changes, we observed paving-stone-like cells in both culture systems (Figures 1(a) and 1(b)). The cells were firmly attached to the Matrigel-coated PET membrane and reached a confluent state after 10 days of culture, in vitro (Figures 1(c) and 1(d)). After air-lifting for a week, COMECs in both the LNCs and 3T3 groups formed stratified structures (Figures 1(e) and 1(f)).

### 3.2. Identification of Differentially Expressed miRNAs

We performed high-throughput sequencing of COMECs cocultured with LNCs or 3T3 cells, and differential miRNA expression with |log2 (fold change)| > 1) and (*P* value <0.05) was analyzed using the *R* package DESeq2. Compared to the 3T3 group, 99 known and 1 newly predicted miRNAs were significantly upregulated, while 101 known and 8 newly predicted miRNAs were significantly downregulated in the LNCs group. According to more stringent criteria, baseMean is greater than 500, |log2 (fold change)| > 1.18, *P* value <0.04, and the top 60 significantly differentially expressed miRNAs (DEmiRNAs; LNCs and 3T3 groups) are given in Table 2. Heatmaps of differentially expressed miRNAs between the LNCs and 3T3 groups are shown in Figure 2(a). All samples were performed three biological replicates separately.

### 3.3. miRNA Target Gene Prediction

We used starBase to predict the target genes of 60 miRNAs with significant differences, and a total of 3000 target genes were predicted. Through a more stringent screening of miRNA expression levels, differential fold change, and *P* values, 14 miRNAs with significant differences (7 upregulated and 7 downregulated) and their target genes were finally screened, as given in Table 3. The 14 miRNAs screened above were used for target gene prediction, and a miRNA-mRNA regulatory network was constructed. There is a close regulatory relationship between miRNA and target genes. The same miRNA can regulate multiple genes, and similarly, the same gene may be regulated by multiple miRNAs. Many of these target genes have been reported to be closely related to angiogenesis, such as CREBBP, MAP3K13, NOX4, PANK3, VEGFB, and MAPK7 (Figure 2(d)).

### 3.4. KEGG and GO Pathway Analyses

To explore the potential functions of these DEmiRNAs, GO and KEGG pathway enrichment analyses were performed. The KEGG pathway analysis revealed that the target genes of DEmiRNAs mainly involved with the VEGF, HIF-1, melanogenesis, Ras, synaptic vesicle cycle, NF-kappa *β*, PI3K-Akt, Notch, and MAPK signaling pathway (Figure 2(b)). In addition, the GO analysis revealed that the target genes of DEmiRNAs were mostly involved in biological processes, such as signal release, cell surface receptor signaling pathway involved in cell-cell signaling, regulation of vesicle-mediated transport, positive regulation of MAPK cascade, and dephosphorylation. Other target genes codified for cellular components, such as presynaptic and postsynaptic ones, and for effectors of specific molecular functions, including metal ion transmembrane transporter activity, monovalent inorganic cation transmembrane transporter activity, positive regulation of cell migration, and passive transmembrane transporter activity (Figure 2(c)).

### 3.5. Relationship between miRNA Expression and KEGG Pathway

In order to better understand the relationship between KEGG pathways and miRNAs expression, we constructed regulatory network of them. First, the target genes of the miRNA were predicted, and then, the corresponding target genes were enriched with KEGG, and finally, the miRNA and KEGG were linked together. The 14 differentially expressed miRNAs were analyzed, and they were finally found that in addition to rno-miR-379-5p, the other 13 miRNAs were involved in the regulation of angiogenesis-related KEGG pathways, such as VEGF, HIF-1, Ras, NF-kappa *β*, PI3K-Akt, and Notch, and MAPK signaling pathway (Figure 2(e)).

### 3.6. Isolation and Extraction of Exosomes from the Supernatant of Cocultured Cell

To explain the stronger inhibition of corneal angiogenesis by COMECs cocultured with LNCs (LNCs group) than those cocultured with 3T3 (3T3 group), we collected cell supernatants from the transwell culture systems and performed exosomes isolation and identification and RNA extraction. The characterization of exosomes from COMECs is shown in Figure 3(a). Results of translucent electron microscope observation showed that the vesicles derived from COMECs of the LNCs and 3T3 groups displayed similar shapes and sizes (Figures 3(b) and 3(c)), ranging from 50 to 150 nm, with the majority presenting <100 nm diameter in both the groups (Figures 3(d) and 3(e)). To further characterize the vesicles, Western blotting was performed to detect the exosome-specific antigen molecules CD9 and TSG101. The results indicated that all samples expressed these markers, and there were no significant differences in the total protein content between the COMECs of the LNCs and 3T3 groups. These findings show that the cell supernatant derived from COMECs cocultures with LNCs and 3T3 cells is rich in exosomes, which indicates that the intercellular communication between those cells was very active.

### 3.7. Measurement of Expression Levels of Candidate miRNAs Using RT-qPCR

Sequencing of the cell lines revealed that the expression levels of rno-miR-200a-5p, rno-miR-204-5p, rno-miR-126a-3p, rno-miR-192-5p, rno-miR-211-5p, rno-miR-143-3p, and rno-miR-184 were significantly higher in the LNCs group than the 3T3 group. Following, we performed RT-qPCR measurement of exosomal miRNA levels on the candidate miRNAs, and the results showed a similar trend in the expression levels of most miRNAs obtained from the supernatant of COMECs cocultured with LNCs or 3T3 cells had a similar trend in exosomes (Figure 4(a)). Meanwhile, seven miRNAs were significantly downregulated in the LNCs group compared to 3T3 group in the cells, and three of them, rno-miR-23a-3p, rno-miR-379-5p, and rno-miR-127-5p, were also significantly downregulated in exosomes, while rno-miR-24-3p, rno-miR-434-5p, rno-miR-483-5p, and rno-miR-541-5p were not (Figure 4(b)). All samples of exosomes were performed in three biological replicates. Altogether, these results suggest that the signal transduction of specific miRNAs between cells through exosomes may be an important factor for the inhibition of angiogenesis by LNCs nourished COMECs.

## 4. Discussion

Currently, autologous limbal tissue/stem cell transplantation is the most established treatment for LSCD, which shows a favorable and stable therapeutic effect; however, this procedure cannot be used in patients with binocular LSCD. Clinical observations revealed that the most severe LSCD often involved both eyes, forcing ophthalmologists to choose allogeneic sources of corneal tissue or cells for treatment [22]. Nonetheless, this option is accompanied by a high risk of immune rejection and requires long-term adjuvant therapy using immunosuppressants, thus limiting the clinical benefits of the treatment. The development of regenerative medicine and stem cell therapy has brought new hope for patients with bilateral LSCD. OMECs are derived from the same ectoderm as corneal epithelial cells and can be used as “seeds” to treat bilateral LSCD, greatly reducing the risk of immune rejection after surgery [11]. As an alternative to allogeneic cultivated limbal epithelial transplantation, COMET promotes corneal epithelialization, suppresses inflammatory reaction, promotes corneal ulcer healing, prevents corneal perforation, and restores residual limbal stem cell/corneal epithelial cell function [3]. However, the postoperative peripheral corneal neovascularization hindered the wide application of this technique. Preliminary studies have shown that LNCs, one of the components of the limbal microenvironment, could participate in the in vitro culture of OMECs as feeders, and inhibit the regeneration of peripheral corneal neovascularization after COMET.

In this study, we performed intracellular miRNA sequencing on COMECs in two coculture systems, one with LNCs and another with 3T3 cells, and found that in the different groups of COMECs, compared to the 3T3 group, 99 known and 1 newly predicted miRNAs were significantly upregulated while 101 known and 8 newly predicted miRNAs were significantly downregulated in the LNCs group. Then, we wonder whether these are the reasons for the different situation of peripheral corneal neovascularization after COMET. Previous studies suggested that miRNAs play a key role in inhibiting angiogenesis. miR-184 exhibited angiostatic properties via regulation of Akt and VEGF signaling pathways [23]. circFOXP1 can promote angiogenesis by regulating the miR-127-5p/CDKN2AIP signaling pathway in osteosarcoma [24]. In addition, miR-200 inhibits angiogenesis through direct and indirect mechanisms by targeting interleukin-8 and C-X-C motif chemokine ligand 1 [25]. The prediction of the target genes of 60 miRNAs showed significant differences, and a total of 3000 target genes were identified.

The KEGG pathway analysis revealed that the target genes of the identified DEmiRNAs were mainly associated with the synaptic vesicle cycle, aldosterone-regulated sodium reabsorption, phosphatidylinositol signaling system, melanogenesis, long-term potentiation, oxytocin signaling pathway, MAPK signaling pathway, and regulation of actin cytoskeleton. These KEGG pathways are closely related to angiogenesis [26, 27]. In addition, the GO analysis revealed that the target genes of DEmiRNAs were enriched in several biological processes, molecular functions, and cellular components, such as signal release, cell surface receptor signaling pathway involved in cell-cell signaling, regulation of vesicle-mediated transport, MAPK, dephosphorylation, presynaptic and postsynaptic components, metal ion transmembrane transporter activity, monovalent inorganic cation transmembrane transporter activity, positive regulation of cell migration, and passive transmembrane transporter activity.

The only difference between the two coculture systems was the feeder; therefore, the differences in miRNA expression between the two groups of COMEC cells might be determined by the cell type used as feeder. Exosomes are carriers for material exchange and signal transduction between cells [28], and they contain proteins, RNAs, and miRNAs [29]. Our data suggest that the transduction of exosomes between cells might lead to the alterations in gene expression observed between LNCs and 3T3 groups. In order to investigate how feeder cells affected COMECs, we isolated exosomes and extracted total RNA from the cell supernatants of the two coculture systems. The electron microscopy study and nanoparticle tracking analysis (NTA) and Western blot analyses revealed that the cell supernatants contained a large number of exosomes. Further characterization of the miRNAs contained in the exosomes by qRT-PCR showed that the expression trend of most miRNAs in exosomes is consistent with that observed in COMECs. These results suggest that the differences in miRNA expression affecting COMECs were introduced by the feeder via exosomes. In addition, some miRNAs showed uncorrelated expression trends in exosomes and COMECs, such as rno-miR-24-3p, rno-miR-434-5p, rno-miR-483-5p, and rno-miR-541-5p; which were not significantly different in the exosomes isolated from the two coculture systems. These results may be attributed to the fact that the miRNAs and other macromolecules encapsulated in the exosomes affect the expression of additional miRNAs after entering COMECs. Therefore, our data suggest that the phenotypic alterations observed in COMECs result from a series of regulatory effects that take place after exosome signal transduction.

## 5. Conclusions

In summary, this study revealed that during the coculture of LNCs and OMECs, LNCs released exosomes carrying miRNAs that were transferred to the OMECs, thereby inhibiting the angiogenesis function of OMECs. Our data provide a new research direction and theoretical basis for the inhibition of corneal angiogenesis after COMET and suggests that coculturing with LNCs may inhibit corneal angiogenesis after COMET and optimize its therapeutic effect. Future studies are required to further characterize the specific mechanisms mediating exosome regulation of gene expression.

## Figures and Tables

**Figure 1:** Isolation of OMECs and coculture with feeder cells. (a) OMECs+3T3 coculture for 3 days. (b) OMECs + LNC coculture for 3 days. (c) OMECs + 3T3 coculture for 10 days. (d) OMECs + LNC coculture for 10 days. Stratified COMEC sheets cocultured with 3T3 cells (e) and LNCs (f) had 3-4 layers after air-lifting for one week.

**Figure 2:** Identification of differentially expressed miRNAs and the related KEGG and GO pathways enrichment of target genes. (a) Heatmaps of differentially expressed miRNAs between the LNCs and 3T3 groups. (b) KEGG pathway enrichment analyses of differentially expressed miRNAs. (c) GO pathway enrichment analysis of differentially expressed miRNAs. (d) miRNA-mRNA regulatory network with significant differences. (e) Relationship between the KEGG pathways and miRNAs with significant differences. All samples were performed two biological replicates separately.

**Figure 3:** Identification of exosomes from the supernatant of COMECs cocultured with LNCs or 3T3 cells separately. (a) Western blot identification of LNCs and 3T3 using exosome-specific antigen molecules CD9 and TSG101. (b) Identification of exosomes of 3T3 and (c) LNCs by a translucent electron microscope. (d) Identification the size range of exosomes on 3T3 and (e) on LNCs through NTA.

**Figure 4:** Measurement of expression levels of candidate miRNAs using RT-qPCR in exosomes. (a) Seven exosomal miRNAs significantly upregulated in LNCs compared to 3T3. (b) Three exosomal miRNAs significantly downregulated in LNCs compared with 3T3. All samples were performed two biological replicates separately.

**Table 1:** Primer sequences of 14 miRNAs.

miRNA ID	Primer	Sequence (5′-3′)
rno-miR-204-5p	rno-miR-204-5p-F	CGCGTTCCCTTTGTCATCCT
	rno-miR-204-5p-R	AGTGCAGGGTCCGAGGTATT
	rno-miR-204-5p-URP	GTCGTATCCAGTGCAGGGTCCGAGGTATTCGCACTGGATACGACAGGCAT

rno-miR-184	rno-miR-184-F	CGCGTGGACGGAGAACTGAT
	rno-miR-184-R	AGTGCAGGGTCCGAGGTATT
	rno-miR-184-URP	GTCGTATCCAGTGCAGGGTCCGAGGTATTCGCACTGGATACGACACCCTT

rno-miR-211-5p	rno-miR-211-5p-F	CGCGTTCCCTTTGTCATCCT
	rno-miR-211-5p-R	AGTGCAGGGTCCGAGGTATT
	rno-miR-211-5p-URP	GTCGTATCCAGTGCAGGGTCCGAGGTATTCGCACTGGATACGACAGGCAA

rno-miR-126a-3p	rno-miR-126a-3p-F	CGCGTCGTACCGTGAGTAAT
	rno-miR-126a-3p-R	AGTGCAGGGTCCGAGGTATT
	rno-miR-126a-3p-URP	GTCGTATCCAGTGCAGGGTCCGAGGTATTCGCACTGGATACGACCGCATT

rno-miR-143-3p	rno-miR-143-3p-F	CGCGTGAGATGAAGCACTGT
	rno-miR-143-3p-R	AGTGCAGGGTCCGAGGTATT
	rno-miR-143-3p-URP	GTCGTATCCAGTGCAGGGTCCGAGGTATTCGCACTGGATACGACTGAGCT

rno-miR-23a-3p	rno-miR-23a-3p-F	GCGATCACATTGCCAGGG
	rno-miR-23a-3p-R	AGTGCAGGGTCCGAGGTATT
	rno-miR-23a-3p-URP	GTCGTATCCAGTGCAGGGTCCGAGGTATTCGCACTGGATACGACGGAAAT

rno-miR-379-5p	rno-miR-379-5p-F	GCGCGTGGTAGACTATGGAA
	rno-miR-379-5p-R	AGTGCAGGGTCCGAGGTATT
	rno-miR-379-5p-URP	GTCGTATCCAGTGCAGGGTCCGAGGTATTCGCACTGGATACGACCCTACG

rno-miR-200a-5p	rno-miR-200a-5p-F	CAUCUUACCGGACAGUGCUGG
	rno-miR-200a-5p-R	AGTGCAGGGTCCGAGGTATT
	rno-miR-200a-5p-URP	GTCGTATCCAGTGCAGGGTCCGAGGTATTCGCACTGGATACGACGACCTG

rno-miR-192-5p	rno-miR-192-5p-F	CUGACCUAUGAAUUGACAGCC
	rno-miR-192-5p-R	AGTGCAGGGTCCGAGGTATT
	rno-miR-192-5p-URP	GTCGTATCCAGTGCAGGGTCCGAGGTATTCGCACTGGATACGACGGAACT

rno-miR-541-5p	rno-miR-541-5p-F	CGAAGGGATTCTGATGTTGGT
	rno-miR-541-5p-R	AGTGCAGGGTCCGAGGTATT
	rno-miR-541-5p-URP	GTCGTATCCAGTGCAGGGTCCGAGGTATTCGCACTGGATACGACAGTGTG

rno-miR-483-5p	rno-miR-483-5p-F	CGCGAAGACGGGAGAAGAGA
	rno-miR-483-5p-R	AGTGCAGGGTCCGAGGTATT
	rno-miR-483-5p-URP	GTCGTATCCAGTGCAGGGTCCGAGGTATTCGCACTGGATACGACCTCCCT

rno-miR-127-5p	rno-miR-127-5p-F	CGCTGAAGCTCAGAGGGCT
	rno-miR-127-5p-R	AGTGCAGGGTCCGAGGTATT
	rno-miR-127-5p-URP	GTCGTATCCAGTGCAGGGTCCGAGGTATTCGCACTGGATACGACAATCAG

rno-miR-24-3p	rno-miR-24-3p-F	GCGTGGCTCAGTTCAGCAG
	rno-miR-24-3p-R	AGTGCAGGGTCCGAGGTATT
	rno-miR-24-3p-URP	GTCGTATCCAGTGCAGGGTCCGAGGTATTCGCACTGGATACGACCTGTTC

rno-miR-434-5p	rno-miR-434-5p-F	GCGAGCTCGACTCATGGTTT
	rno-miR-434-5p-R	AGTGCAGGGTCCGAGGTATT
	rno-miR-434-5p-URP	GTCGTATCCAGTGCAGGGTCCGAGGTATTCGCACTGGATACGACTGGTTC

**Table 2:** The top 60 significantly differentially expressed miRNAs.

miRNA ID	BaseMean	log2FoldChange	*P* value	Padj	Direction
rno-miR-184	5018754.403	8.35486	1.6E-146	2.8E-144	Up
rno-miR-21-5p	139245.3834	2.348338	5.87E-21	9.87E-20	Up
rno-miR-200b-3p	49759.61134	1.939218	1.06E-06	4.37E-06	Up
rno-miR-204-5p	46858.87015	12.96147	0	0	Up
rno-miR-26a-5p	38639.14475	1.282148	9.71E-07	4.05E-06	Up
rno-miR-143-3p	38026.17625	3.940324	1.32E-45	5.72E-44	Up
rno-miR-30d-5p	37783.14552	1.579329	3.43E-07	1.53E-06	Up
rno-miR-30a-5p	31780.68609	1.164141	4.84E-11	3.45E-10	Up
rno-let-7g-5p	21746.5107	1.024793	0.009549	0.019743	Up
rno-miR-23a-3p	17257.68677	−2.17059	3.33E-71	3.47E-69	Down
rno-miR-148a-5p	15005.61924	−1.55774	3.47E-05	0.000113	Down
rno-miR-200a-3p	14699.09577	1.168533	0.006848	0.014866	Up
rno-miR-24-3p	13910.08088	−1.54013	3.33E-11	2.44E-10	Down
rno-miR-200a-5p	13458.89538	2.128498	8.48E-07	3.59E-06	Up
rno-miR-127-3p	12045.02124	−3.82274	1.97E-48	9.31E-47	Down
rno-miR-99b-5p	10484.418	1.013676	3.16E-09	1.81E-08	Up
rno-miR-24-2-5p	6441.491879	−2.0134	6.15E-06	2.22E-05	Down
rno-miR-100-5p	6062.273033	1.341755	4.18E-15	4.84E-14	Up
rno-miR-181a-5p	5356.592531	2.317662	1.1E-14	1.24E-13	Up
rno-miR-192-5p	4361.106614	2.829028	1.9E-11	1.48E-10	Up
rno-miR-101a-3p	3806.813811	1.98834	1.62E-21	2.91E-20	Up
rno-miR-30e-5p	3739.554912	1.206808	3.78E-10	2.49E-09	Up
rno-miR-125b-5p	3717.954371	1.720303	1.15E-13	1.13E-12	Up
rno-miR-185-5p	3583.899727	−1.40718	0.000787	0.002102	Down
rno-miR-211-5p	3450.975784	6.508208	8E-303	2.1E-300	Up
rno-miR-126a-3p	3304.770861	4.185799	6.05E-18	8.76E-17	Up
rno-miR-27a-5p	3111.57102	2.785614	2.19E-72	2.86E-70	Up
rno-miR-541-5p	3109.566931	−5.59168	7.22E-61	4.18E-59	Down
rno-miR-30e-3p	2761.433396	1.395479	2.5E-11	1.92E-10	Up
rno-miR-379-5p	2755.226093	−2.75231	1.1E-29	3.02E-28	Down
rno-miR-134-5p	2689.526317	−5.61534	4.29E-27	1.06E-25	Down
rno-miR-676	2491.32323	1.456927	9.67E-14	9.69E-13	Up
rno-miR-361-3p	2095.636071	1.61435	2.31E-39	8.03E-38	Up
rno-let-7e-5p	1657.170086	1.070053	3.1E-14	3.37E-13	Up
rno-miR-181d-5p	1605.480694	−1.46868	1.58E-05	5.47E-05	Down
rno-miR-128-3p	1557.649722	1.502977	1.52E-11	1.23E-10	Up
rno-miR-1839-5p	1446.486591	−1.18747	1.38E-09	8.37E-09	Down
rno-miR-29a-3p	1416.848906	2.1861	4.97E-24	9.6E-23	Up
rno-miR-181b-5p	1202.845297	1.40078	5.29E-06	1.94E-05	Up
rno-miR-125a-5p	1099.615693	1.344694	5.91E-18	8.76E-17	Up
rno-miR-146a-5p	1097.734821	−1.43583	8.23E-10	5.23E-09	Down
rno-miR-98-5p	1047.460758	−1.95831	6.92E-08	3.4E-07	Down
rno-miR-483-5p	979.822134	−6.48039	6.9E-27	1.64E-25	Down
rno-miR-149-5p	931.8865694	−2.01717	6.3E-12	5.38E-11	Down
rno-let-7d-3p	864.1565244	−1.2181	1.53E-11	1.23E-10	Down
rno-miR-872-5p	826.8599798	1.072442	0.008888	0.018539	Up
rno-miR-652-3p	644.1237189	−1.71998	4.2E-07	1.82E-06	Down
rno-miR-6329	589.9848789	2.025303	1.97E-16	2.57E-15	Up
rno-miR-674-3p	565.9663909	2.451183	2.4E-10	1.65E-09	Up
rno-miR-341	550.3226309	−5.30664	3.05E-62	2.65E-60	Down
rno-miR-582-3p	478.5805945	1.826463	3.75E-14	3.99E-13	Up
rno-miR-127-5p	419.1005227	−4.43715	5.07E-25	1.1E-23	Down
rno-miR-125b-1-3p	418.2645815	3.015164	2.26E-45	9.06E-44	Up
rno-miR-434-5p	412.8655617	−3.7971	1.56E-61	1.16E-59	Down
rno-miR-10b-5p	389.7694199	−2.29215	4.03E-19	6.18E-18	Down
rno-miR-3559-5p	389.5237485	2.053502	5.86E-07	2.5E-06	Up
rno-miR-370-3p	376.074973	−5.22176	2.01E-32	5.82E-31	Down
rno-miR-199a-3p	366.7346349	1.799773	8.54E-08	4.16E-07	Up
rno-miR-30c-5p	5925.397	0.889268	0.000509	0.001404	No
rno-miR-31a-5p	1222.205	0.877971	7.07E-09	3.84E-08	No

**Table 3:** Expression of 14 miRNAs (7 upregulated and 7 downregulated).

miRNA id	BaseMean	log2 fold change	*P* value	*P* adj	Direction
rno-miR-204-5p	71888.2488	12.98945771	2.5424E-136	1.1898E-133	Up
rno-miR-184	7674728.425	8.422128575	1.57194E-63	3.67833E-61	Up
rno-miR-211-5p	5288.532219	6.612171345	1.24127E-48	1.93638E-46	Up
rno-miR-126a-3p	5072.286489	4.391974046	3.58891E-12	7.99813E-11	Up
rno-miR-200a-5p	20257.28133	2.32478216	8.48815E-05	0.00052966	Up
rno-miR-143-3p	57942.39362	4.102096163	1.66877E-16	6.50819E-15	Up
rno-miR-192-5p	6606.603299	3.013336244	1.78547E-07	2.32111E-06	Up
rno-miR-23a-3p	24761.14809	−2.050920428	2.78616E-06	2.46023E-05	Down
rno-miR-379-5p	3850.748446	−2.59440525	9.89696E-08	1.40357E-06	Down
rno-miR-541-5p	4529.097341	−5.523992152	3.09589E-27	3.62219E-25	Down
rno-miR-483-5p	1472.191185	−6.4539066	2.98102E-21	1.99302E-19	Down
rno-miR-127-5p	619.8571292	−4.37982954	7.89498E-14	2.17344E-12	Down
rno-miR-24-3p	19766.72861	−1.390058699	0.003504021	0.012614475	Down
rno-miR-434-5p	585.1719062	−3.665678358	2.74024E-13	7.12462E-12	Down

## Data Availability

The datasets used and analyzed during the current study are available from the corresponding author upon request.
